The article "An Efficient Stacked Deep Transfer Learning Model for Automated Diagnosis of Lyme Disease" was retracted in 2023. Reasons: unreliable results or conclusions; concerns about the data; concerns about the results or conclusions; concerns about the peer review.

# An Efficient Stacked Deep Transfer Learning Model for Automated Diagnosis of Lyme Disease

**DOI:** 10.1155/2022/2933015

**Published:** 2022-02-28

**Authors:** Ahmad Ali AlZubi, Shailendra Tiwari, Kuldeep Walia, Jazem Mutared Alanazi, Firas Ibrahim AlZobi, Rohit Verma

**Affiliations:** ^1^Computer Science Department, Community College, King Saud University, Riyadh, Saudi Arabia; ^2^Department of Computer Science and Engineering, Thapar Institute of Engineering & Technology, Patiala, India; ^3^Sri Guru Granth Sahib World University, Fatehgarh Sahib, Punjab, India; ^4^Department of Information Systems and Networks, Faculty of Information Technology, The World Islamic Sciences & Education University, Amman, Jordan; ^5^School of Computing, National College of Ireland, Dublin, Ireland

## Abstract

Lyme disease is one of the most common vector-borne infections. It typically causes cardiac illnesses, neurologic illnesses, musculoskeletal disorders, and dermatologic conditions. However, most of the time, it is poorly diagnosed due to many similarities with other diseases such as drug rash. Given the potentially serious consequences of unnecessary antimicrobial treatments, it is essential to understand frequent and uncommon diagnoses that explain symptoms in this population. Recently, deep learning models have been used for the diagnosis of various rash-related diseases. However, these models suffer from overfitting and color variation problems. To overcome these problems, an efficient stacked deep transfer learning model is proposed that can efficiently distinguish between patients infected with Lyme (+) or infected with other infections. 2^nd^ order edge-based color constancy is used as a preprocessing approach to reduce the impact of multisource light from images acquired under different setups. The AlexNet pretrained learning model is used for building the Lyme disease diagnosis model. To prevent overfitting, data augmentation techniques are also used to augment the dataset. In addition, 5-fold cross-validation is also used. Comparative analysis indicates that the proposed model outperforms the existing models in terms of accuracy, f-measure, sensitivity, specificity, and area under the curve.

## 1. Introduction

Lyme disease is one of the most common vector-borne infections, generally due to one of the three pathogenic genospecies of the spirochete Borrelia [1, 2]. It typically causes cardiac illnesses, neurologic illnesses, musculoskeletal disorders, dermatologic conditions, etc. [3, 4]. However, most of the time, it is poorly diagnosed due to many similarities with other diseases such as drug rash [5], pityriasis rosea rash [6], and ringworm [7].  Figure 1 shows the example of Lyme disease along with other similar diseases. It is clearly found that the drug rash, pityriasis rosea rash, and ringworm visually seem to be similar and so many times, Lyme disease is either underdiagnosed or overdiagnosed.

The article "An Efficient Stacked Deep Transfer Learning Model for Automated Diagnosis of Lyme Disease" was retracted in 2023. Reasons: unreliable results or conclusions; concerns about the data; concerns about the results or conclusions; concerns about the peer review.

Overdiagnosis or underdiagnosis of Lyme disease leads to unnecessary antibiotic treatments. Numerous problems and adverse consequences because of medicines being given to patients longer than recommended, needless antibiotics, or unusual therapies for Lyme disease were reported, like cholecystitis, catheter-associated bloodstream infection, clots from venous catheters, *Clostridioides difficile* infections, and death. Given the potentially serious consequences of unnecessary antimicrobial treatments, it is essential to understand frequent and uncommon diagnoses that explain symptoms in this population [2–4].

Therefore, it is required to build such a framework or model which can clearly distinguish among patients infected with Lyme (+) or infected with other infections. Recently, the imaging dataset of Lyme patients has been published on the Kaggle website [8]. Many researchers have utilized it for distinguishing between Lyme infections and infections with other rashes using deep learning models. However, these models suffer from the overfitting problem. Also, suitable preprocessing techniques are required to improve the quality of images under consideration to achieve efficient results. To overcome these problems, in this paper, an efficient stacked deep transfer learning model is proposed to classify Lyme patients.

The main contributions of this paper are as follows:

- An efficient stacked deep transfer learning model is proposed to classify Lyme patients
- 2^nd^ order edge-based color constancy is used as a preprocessing approach to reduce the impact of multisource light from images acquired under different setups
- The AlexNet pretrained learning model is used
- Data augmentation techniques are also used to augment the dataset

The remaining paper is organized as follows: Section 2 presents the literature work, Section 3 presents the proposed model, Section 4 discusses various experimental results, and Section 5 concludes the paper.

## 2. Related Work

In [9], an ensemble deep learning pipeline (EDLP) was designed by using the 34-layer ResNet model. ResNet was used to extract the features from the limited skin disease dataset. Eleven skin conditions were classified. It has achieved 91.7% precision and 92.55% recall, respectively. In [10], skin cancer was evaluated from the rashes. A convolutional neural network (CNN) was utilized to predict images of rashes or skin cancer. It has achieved an accuracy of 80.2% for 20 epochs. In [11], a mobile-enabled expert system named i-Rash was designed for the diagnosis of inflammatory skin lesions. It can predict the given image as psoriasis, eczema, acne, and healthy. i-Rash was trained using pretrained SqueezeNet.

The article "An Efficient Stacked Deep Transfer Learning Model for Automated Diagnosis of Lyme Disease" was retracted in 2023. Reasons: unreliable results or conclusions; concerns about the data; concerns about the results or conclusions; concerns about the peer review.

In [12], a lightweight attention-based deep learning model (LWADL) was designed to predict eleven skin diseases. LWADL achieved better accuracy as compared to VGG19, VGG16, ResNet50, and InceptionV3. In [13], a UNet-based dense CNN (UNet-dCNN) model was designed. MobileNetV2 was also used to achieve better results. It was utilized for histopathological image-based skin cancer diagnosis. It has shown an average accuracy of 87.7%. In [14], a multitask deep learning model was designed. It was utilized for automatic analysis and classification of skin lesions. A focal loss and a Jaccard distance-based loss function were designed. A three-phase joint training approach was used to assure significant feature learning.

In [15], a pretrained ResNet-50 model was utilized for the classification of melanoma. Ensemble learning was also considered to obtain better results. In [16], a fully automated deep ensemble model (FADEM) was designed for lesion boundary segmentation. DeeplabV3+ and Mask R-CNN were ensembled and tested on the ISIC-2017 dataset. FADEM has achieved specificity and sensitivity of 97.94% and 89.93%, respectively. In [17], ensembling of CNN models was achieved by integrating with a test-time regularly spaced shifting. The proposed ensemble model was used for the classification of skin lesions. In [18], an adaptive dual attention module-based CNN model was designed for the segmentation of skin lesions. The proposed model has shown better performance during the computation of potential features in classifying the skin lesions' boundary.

From the existing literature, it is found that the existing models suffer from overfitting and hyperparameter tuning problems. In addition, preprocessing techniques are required to reduce the impact of multiple light sources on the images. Also, none of the researchers have focused on the diagnosis of Lyme disease. Therefore, in this paper, an efficient model is designed to achieve better results.

## 3. Proposed Methodology

This section discusses the proposed methodology. Initially, the obtained images are improved by using the 2^nd^ order edge color constancy. Thereafter, a ResNet-based model is trained to achieve better results [18].  Figure 2 shows the proposed automated Lyme disease diagnosis model. It clearly shows that the proposed model is decomposed into three phases, i.e., data augmentation, 2^nd^ order edge-based color constancy, and an AlexNet-based pretrained model for extracting the features which are used for the classification using fully connected layers. To achieve regularization and to prevent overfitting, dropouts are also used. Binary cross-entropy is used as a loss function.

The article "An Efficient Stacked Deep Transfer Learning Model for Automated Diagnosis of Lyme Disease" was retracted in 2023. Reasons: unreliable results or conclusions; concerns about the data; concerns about the results or conclusions; concerns about the peer review.

### 3.1. Color Constancy

Color constancy has the ability to restore the impact infected multiple light sources. Thus, the obtained images are independent of colors of the light source. In this paper, a 2^nd^ order-edge based color constancy approach is used. It states that the distribution of color derivatives exhibits the principal dissimilarity in the direction of a light source [18]. Minkowski's norm is then applied to the computed derivatives to predict the direction of a light source [19, 20]. A step-by-step algorithm for the 2^nd^ edge-based color constancy is presented in Algorithm 1.

### 3.2. Proposed ResNet Model

Residual network (ResNet) is a well-known pretrained model used as a backbone for classifying many imaging datasets. It allowed us to successfully build an enormously deep model with more than 150 layers. Before ResNet, the existing models suffered from vanishing gradients whenever we tried to train them deeply. It has achieved better results with the help of skip connections. It prevents the vanishing gradient problem by using a substitute shortcut route for the gradient to flow through. It allows the model to build an identity function that assures the topmost layer will achieve better performance, the same as the lower layer.

Figure 3 shows the ResNet model in the paper. Initially, the images obtained from the color constancy model are utilized for building the trained model. It utilizes various convolution layers, followed by ReLU, normalization, and pooling operations. After using 5 convolution layers, a fully connected layer is utilized along with ReLU and dropouts. Finally, after using three fully connected layers, the softmax function is used to obtain the results.

## 4. Experimental Analysis

The experiments for the proposed model are performed on the online MATLAB 2021a using a benchmark Kaggle dataset. Comparisons are also performed by considering the competitive models. In addition, we have also validated the proposed model with and without considering the 2nd order edge-based color constancy.  Table 1 demonstrates the hyperparameter setting of the proposed model.

### 4.1. Dataset

In this paper, the Lyme disease (Silent Epidemic) dataset [8] obtained from Kaggle is used for experimental purposes. It composes images of the erythema migrans, referred to as bull's eye rash. It is one of the utmost protuberant signs of Lyme disease. The dataset also includes other kinds of rashes that may be often confused with Lyme disease by medical staff. For training, there are 206 Lyme (-ve) and 151 Lyme (+ve) images available. For testing, there are 51 Lyme (-ve) and 36 Lyme (+ve) images available.

The article "An Efficient Stacked Deep Transfer Learning Model for Automated Diagnosis of Lyme Disease" was retracted in 2023. Reasons: unreliable results or conclusions; concerns about the data; concerns about the results or conclusions; concerns about the peer review.

Therefore, data augmentation is used to augment the dataset. Since the obtained images were captured using different machines under different light sources, using these images directly for diagnosis may result in poor performance of the model. Therefore, in this paper, to prevent the effect of multiple light sources, color constancy is used. It can restore the impact of color light sources from the images to achieve better performance of the models.

### 4.2. Training and Validation Analysis

Figure 4 shows the training and validation analysis of the proposed model without the use of 2^nd^ order edge-based color constancy. It clearly shows that the proposed model has achieved 95.71% validation accuracy. But also, it is found that the proposed model suffers from the overfitting issue since the training accuracy is 100%. Therefore, still, there is room for improvement in it.

Figure 5 shows the training and validation accuracy of the proposed model with 2^nd^ order edge-based color constancy. It is found that the proposed model with color constancy achieves 98.69% validation accuracy. Therefore, the proposed model is least affected by the overfitting problem. Besides, the validation accuracy of the proposed model has shown better convergence speed than in the results shown in Figure 4.

### 4.3. Confusion Matrix Analysis

Confusion matrix analyses are widely accepted to compute the performance of the various classification models. It utilizes the concepts of true positive (TP), true negative (TN), false positive (FP), and false negative (FN) that can be computed using the actual and predicted classes.

Figure 6 shows the confusion matrix of the proposed model without the use of 2^nd^ order edge-based color constancy. It is found that without the use of color constancy, the proposed model achieves an average accuracy of 95.7%. It is found that this model has achieved better results, but with a 4.3% error rate.

Figure 7 demonstrates the confusion matrix analysis of the proposed model with 2^nd^ order edge-based color constancy. It is found that the proposed model has achieved 98.7% accuracy, which is 2.0% better than the proposed model without the use of 2^nd^ order edge-based color constancy (EBCC). There are only 7 cases that are poorly classified by the proposed model, compared to 23 in the model with the use of 2^nd^ order edge-based color constancy.

### 4.4. Discussion

This section presents the discussion of the proposed and competitive models when they are applied to the Lyme disease dataset. The hyperparameters of the competitive models are obtained from their published papers. These competitive models are CNN [10], EDLP [9], SqueezeNet [11], LWADL [12], Unet-dCNN [13], ResNet-50 [15], FADEM [16], and Ensemble CNN [17].  Table 2 demonstrates the testing analysis of the proposed and competitive models. It is found that the proposed model achieves remarkably better performance than the competitive models. Bold values represent the better-performing model. The proposed model has achieved an average improvement in terms of accuracy, f-measure, sensitivity, specificity, and area under the curve (AUC) as 2.9787%, 2.7891%, 3.0875%, 2.1578%, and 2.1579%, respectively.

The article "An Efficient Stacked Deep Transfer Learning Model for Automated Diagnosis of Lyme Disease" was retracted in 2023. Reasons: unreliable results or conclusions; concerns about the data; concerns about the results or conclusions; concerns about the peer review.

It is found that the proposed model achieves remarkable performance for Lyme disease. Therefore, the proposed model can be used for real-time diagnosis of Lyme disease and can help doctors treat patients with the correct medicines.

## 5. Conclusion

This paper proposes an efficient stacked deep transfer learning model that can efficiently distinguish between patients infected with Lyme (+) or infected with other infections. 2^nd^ order edge-based color constancy was used as a preprocessing approach to reduce the impact of multisource light from images acquired under different setups. The AlexNet pretrained learning model was utilized for building the Lyme disease diagnosis model. Data augmentation techniques were also used to augment the dataset. Extensive comparative analyses have shown that the proposed model outperforms the competitive models in terms of accuracy, f-measure, sensitivity, specificity, and AUC of 2.9787%, 2.7891%, 3.0875%, 2.1578%, and 2.1579%, respectively.

## Figures and Tables

**Figure 1:** Images of Lyme disease along with other similar diseases.

**Figure 2:** The proposed automated Lyme disease diagnosis model.

**Figure 3:** The proposed ResNet-based classification architecture for Lyme diagnosis.

**Figure 4:** Training and validation analysis of the proposed model without using the 2^nd^ order edge-based color constancy.

**Figure 5:** Training and validation analysis of the proposed model with 2^nd^ order edge-based color constancy.

**Figure 6:** Confusion matrix analysis of the proposed model without 2^nd^ order edge-based color constancy.

**Figure 7:** Confusion matrix analysis of the proposed model with 2^nd^ order edge-based color constancy.

**Algorithm 1:** Second-order edge-based color constancy algorithm.

**Table 1:** Hyperparameter setting of the proposed model.

Parameter	Value/type
Gradient decay factor	0.9
Squared gradient decay factor	0.99
Epsilon	1.00E-08
Initial learning rate	3.00E-04
Learning rate drop factor	0.1
Learning rate drop period	10
L2 regularization	1.00E-04
Gradient threshold	L2-norm
Maximum epochs	200
Minimum batch size	64
Validation frequency	50

The article "An Efficient Stacked Deep Transfer Learning Model for Automated Diagnosis of Lyme Disease" was retracted in 2023. Reasons: unreliable results or conclusions; concerns about the data; concerns about the results or conclusions; concerns about the peer review.

**Table 2:** Training analyses among the proposed and competitive Lyme rash classification models.

Model	TP	FP	TN	FN	Accuracy	f-measure	Sensitivity	Specificity	AUC
CNN [10]	196	20	294	26	90.4306	91.5032	87.9069	93.3333	91.0679
EDLP [9]	192	24	303	17	89.6551	94.3708	92.4444	92.2330	92.3221
SqueezeNet [11]	194	22	294	26	89.3719	92.1921	87.6777	93.3130	91.1111
LWADL [12]	210	6	295	25	97.0731	92.4471	88.8392	98.0769	94.2164
Unet-dCNN [13]	184	32	297	23	86.0262	92.6282	89.5454	90.0311	89.8336
ResNet-50 [15]	202	14	288	32	93.1372	89.8089	85.5855	95.2702	91.1196
FADEM [16]	195	21	292	28	90.1408	91.3580	87.2727	93.3753	90.8752
Ensemble CNN [17]	195	21	310	10	90.7894	96.633	95.3917	93.1818	94.0952
Proposed without EBCC	197	19	316	4	90.5940	98.6486	97.8609	93.8906	95.3815
Proposed with EBCC	213	3	316	4	98.6111	98.6711	98.1566	99.0000	98.6460

## Data Availability

The used dataset is freely available at https://www.kaggle.com/sshikamaru/lyme-disease-rashes.
